# Expression Pattern and Prognostic Value of EPHA/EFNA in Breast Cancer by Bioinformatics Analysis: Revealing Its Importance in Chemotherapy

**DOI:** 10.1155/2021/5575704

**Published:** 2021-04-22

**Authors:** Zheng Liang, Xu Wang, Kaiti Dong, Xinhua Li, Chenge Qin, Huifang Zhou

**Affiliations:** ^1^Department of Otorhinolaryngology, Tianjin Medical University General Hospital, Tianjin 300052, China; ^2^Department of Breast Oncology, Key Laboratory of Breast Cancer Prevention and Therapy (Ministry of Education), Key Laboratory of Cancer Prevention and Therapy, Tianjin, National Clinical Research Center for Cancer, Tianjin's Clinical Research Center for Cancer, Tianjin Medical University Cancer Institute and Hospital, Tianjin 300060, China

## Abstract

The activities of the ephrin family in breast cancer (BrCa) are complex. Family A receptors (EPHA) and ligands (EFNA) can act as oncogenes or tumor suppressors and are implicated in chemoresistance. Here, we examined the expression pattern and prognostic value of the EPHA/EFNA family in patients with breast cancer, including patients with different subtypes or different chemotherapy cohorts. In the UALCAN database, the mRNA expression of EPHA1, EPHA10, EFNA1, EFNA3, and EFNA4 was significantly higher, whereas that of EPHA2, EPHA4, EPHA5, and EFNA5 was significantly lower in breast cancer tissues than in paracancerous tissues. The transcriptional levels of EPHA/EFNA family members were correlated with intrinsic subclasses of breast cancer. The relationship between EPHA/EFNA and the clinicopathological parameters of BrCa was analyzed using bc-GenExMiner V4.5. EPHA1, EPHA2, EPHA4, EPHA7, EFNA3, EFNA4, and EFNA5 were upregulated in estrogen receptor- (ER-) and progesterone receptor- (PR-) negative tumors, whereas EPHA3, EPHA6, and EFNA1 were upregulated in ER- and PR-positive tumors. EPHA1, EPHA2, EFNA3, and EFNA4 mRNA expression was significantly higher in human epidermal growth factor receptor 2- (HER2-) positive tumors than in HER2-negative tumors. Triple-negative status was positively correlated with EPHA1, EPHA2, EPHA4, EPHA7, EFNA3, EFNA4, and EFNA5 and negatively correlated with EPHA3 and EPHA10 mRNA expression. Genetic alterations of EPHA/EFNA in breast cancer varied from 1.1% to 10% for individual genes, as determined by the cBioPortal database. The Kaplan–Meier plotter indicated that high EphA7 mRNA expression was associated with poor overall survival (OS) and recurrence-free survival (RFS), especially in the HER2 and luminal A subtypes. EFNA4 was predicted to have poor OS and RFS in breast cancers, especially in luminal B, basal-like subtype, and patients treated with adjuvant chemotherapy. High EPHA3 expression was significantly associated with better OS and RFS, especially in the luminal A subtype, but with poor RFS in BrCa patients receiving chemotherapy. Our findings systematically elucidate the expression pattern and prognostic value of the EPHA/EFNA family in BrCa, which might provide potential prognostic factors and novel targets in BrCa patients, including those with different subtypes or treated with chemotherapy.

## 1. Introduction

Breast cancer is the most commonly diagnosed female cancer and the cause of 685,000 cancer mortality in 2020 worldwide [1]. Tumor recurrence and metastasis contribute to the high death rate [2]. Despite extensive research into the treatment of BrCa, chemotherapy resistance is an important issue limiting the efficacy of treatment. Novel biomarkers to predict prognosis or the sensitivity to chemotherapy are urgently needed.

Receptor tyrosine kinases (RTKs) play an important role in a variety of cellular processes in cancer [3]. Ephrins, also known as ephrin ligands, and Eph receptors (Ephs), which are RTKs, are key regulators of physiological and pathological processes involved in development and disease, such as cellular motility, cell repulsion, and cell adhesion [4]. The Ephrin family consists of multiple Ephs and ephrins. Both receptors and ligands are membrane-bound proteins that require direct cell-cell interaction for activation. Eph/ephrin signal transduction occurs not only in the receptor-expressing cell but also in the ligand-expressing cell via bidirectional signaling [5]. The ligands can have a glycosylphosphatidylinositol anchor (A type) or a membrane-spanning protein domain (B type). The receptors are also categorized as A or B according to the type of ligand they bind to. Ephrin family A includes ten receptors named EPHA (1–10) and five ligands designated as EFNA (1–5) [6]. The interaction between ligands and receptors via bidirectional signaling and its involvement in cancer biology are mediated by complex processes [7, 8]. Several Ephrin A (EPHA/EFNA) family members are overexpressed or downregulated in a variety of tumors, suggesting that they act as oncogenes or as tumor suppressors according to the cellular context [9]. Ephrin A family members that are overexpressed in cancer including EFNA1 in melanoma [10]; EPHA2 in prostate cancer [11], nasopharyngeal carcinoma [12], and squamous-cell carcinoma of the head and neck [13]; and EPHA3 in non-small-cell lung cancer [14]. EPHA7 acts as a tumor suppressor in follicular lymphoma and is a potential therapeutic target [15]. EphA2 expression levels are associated with the invasiveness and aggressive behavior of BrCa [16]. The role of EPHA/EFNA as tumor suppressors in breast carcinogenesis was also demonstrated by targeting EPHA2 [17]. EPHA2 regulates the sensitivity to paclitaxel in nasopharyngeal carcinoma via the phosphoinositide 3-kinase/Akt signaling pathway [18]. Cisplatin chemotherapy-induced ERK1/2-RSK1/2-EphA2-GPRC5A signaling is related to acquired chemoresistance in ovarian cancer [19]. Previous findings indicate that EPHA/EFNA family members may serve as biomarkers for predicting prognosis or the response to treatment, which prompted us to analyze the expression pattern and prognostic role of the EPHA/EFNA family in BrCa.

Online databases provide access to a wealth of information, such as microarray RNA chips from the Gene Expression Omnibus (GEO) [20] and RNA sequences from The Cancer Genome Atlas (TCGA) [21]. In this study, we compared the transcriptional levels of EPHA/EFNA in BrCa and paracancerous tissues using the UALCAN database [22]. The relationship between members of the EPHA/EFNA family and clinicopathologic characteristics of BrCa patients was analyzed using breast cancer gene expression miner (bc-GenExMiner) v4.5 [23, 24]. Genetic alterations of EPHA/EFNA family members, including mutations and putative copy number alterations (CNAs), were analyzed in cBioPortal [25]. Moreover, the association of EPHA/EFNA gene expression with clinical outcomes was assessed in patients with BrCa, including patients with different subtypes or those undergoing chemotherapy, using the Kaplan–Meier plotter database [26].

## 2. Methods and Materials

### 2.1. Gene Expression Analysis in UALCAN

UALCAN (http://ualcan.path.uab.edu/) is an online comprehensive and interactive platform based on RNA-seq data and clinical information from TCGA database [22]. In this study, UALCAN was used to investigate the transcriptional levels of EPHA/EFNA family members in primary BrCa tissues and their association with the subtype.

### 2.2. Analysis of the Relationship between EPHA/EFNA and Clinicopathologic Characteristics in Bc-GenExMiner

Bc-GenExMiner v4.5 (http://bcgenex.centregauducheau.fr/BC-GEM), a statistical mining tool of published BrCa transcriptomic data, was used to evaluate the relationship between EPHA/EFNA family members and the clinicopathologic characteristics of BrCa patients, including age, nodal status, estrogen receptor (ER) status, progesterone receptor (PR) status, human epidermal growth factor receptor 2 (HER2) status, lymph node status, triple-negative tumors, and P53 status (sequence). Information on ER, PR, HER2, lymph node status, and pathological grade was not available for all 3,996 patients.

### 2.3. Genetic Alterations Analysis in cBioPortal

OncoPrint is a feature of cBioPortal, an open-source web application that allows researchers to explore and analyze cancer genomic datasets (http://www.cbioportal.org/) [27, 28]. In this study, genetic alterations of EPHA/EFNA family members including mutations and putative CNAs were analyzed. A total of 1084 tumor samples with RNA-seq data on cBioPortal were included in the study.

### 2.4. The Prognostic Value of EPHA/EFNA mRNA Expression in BrCa Patients including Those with Different Subtypes and Undergoing Chemotherapy

The Kaplan–Meier plotter is an online database that facilitates predicting the effect of gene expression on survival in cancer. Sources for the database include GEO, EGA (European Genome-Phenome Archive), and TCGA. This platform, which contains gene expression information and survival data of BrCa patients, was used to perform a meta-analysis to verify the prognostic value of EPHA/EFNA family members for predicting overall survival (OS) and relapse-free survival (RFS). Additional analyses were restricted to cohorts according to subtype and including the patients treated with chemotherapy. Kaplan–Meier survival plots were used to compare the prognosis of all cohorts. Hazard ratios (HRs), 95% confidence intervals (CIs), and log-rank *P* values were calculated and displayed online.

### 2.5. Statistical Analysis

The differential mRNA expression of EPHA/EFNA in BrCa tissues was compared by Student's *t*-test. The log-rank test was used to compare Kaplan-Meier survival plots. A *P* value of <0.05 was considered statistically significant.

## 3. Results

### 3.1. Transcriptional Levels of EPHA/EFNA in BrCa

To evaluate the expression pattern of EPHA/EFNA in BrCa, the transcriptional levels of EPHA/EFNA family members were compared between BrCa and paracancerous tissues using the UALCAN database. As shown in Figure 1, EPHA2 (Figure 1(b), *P* < 0.001), EPHA4 (Figure 1(d), *P* < 0.001), and EPHA5 (Figure 1(e), *P* < 0.001) expression was significantly lower in BrCa tissues than in paracancerous tissues. EPHA1 (Figure 1(a), *P* < 0.001) and EPHA10 (Figure 1(h), *P* < 0.001) expression was significantly higher in BrCa than in paracancerous tissues (Figure 1(f), *P* < 0.001). The expression of EPHA3 (Figure 1(c), *P* = 0.314), EPHA6 (Figure 1(f), *P* = 0.266), and EPHA7 (Figure 1(g), *P* = 0.521) did not differ significantly between BrCa and paracancerous tissues. Analysis of EFNA expression showed that the transcriptional levels of EFNA1 (Figure 1(i), *P* < 0.001), EFNA3 (Figure 1(j), *P* < 0.001), and EFNA4 (Figure 1(k), *P* < 0.001) were significantly higher in BrCa than in paracancerous tissues, whereas the transcriptional level of EFNA5 (Figure 1(l), *P* < 0.001) was significantly lower in BrCa than in paracancerous tissues. EPHA8 and EFNA2 were expressed at markedly low levels according to the UALCAN database, and they were not included in the analysis.

### 3.2. Transcriptional Levels of EPHA/EFNA in Different BrCa Subtypes

The classification of BrCa into subtypes is helpful for predicting the therapeutic response and prognosis of patients [29]. Here, we analyzed the transcriptional levels of EPHA/EFNA family members according to BrCa subtype using the UALCAN database. As shown in Figure 2, EPHA3, EPHA5, EPHA6, and EPHA10 mRNA levels were low in HER2-positive and triple-negative BrCa patients, whereas other EPHA family members did not show this trend. EPHA3, EPHA5, EPHA6, and EPHA10 were expressed at high levels in the luminal subtype (Figures 2(c), 2(e), 2(f), and 2(h)). The highest mRNA expression levels of EFNA were detected in triple-negative tissues except EFNA3, whereas the luminal subtype showed the lowest EFNA mRNA levels (Figures 2(i)–2(l)) except EFNA1. Taken together, these findings indicate that the transcriptional levels of EPHA/EFNA family members are correlated with intrinsic subclasses in BrCa patients.

### 3.3. Association between EPHA/EFNA mRNA Expression and the Clinicopathological Features of Patients with BrCa

We used bc-GenExMiner v4.5 to examine the relationship between EPHA/EFNA and the clinicopathologic characteristics of patients. For the age parameter, EPHA2 (*P* = 0.0002), EPHA3 (*P* < 0.0001), EFNA4 (*P* = 0.0003), and EFNA5 (*P* < 0.0001) were expressed at high levels in patients aged ≤51 years (Table 1). EFNA1 (*P* < 0.0001) and EFNA3 (*P* = 0.0092) were expressed at high levels in older patients, whereas the mRNA expression levels of the other EPHA/EFNA family members were not significantly correlated with age. EPHA2 (*P* = 0.0142) mRNA was higher in BrCa patients with negative lymph nodes than in those with positive lymph nodes, whereas EFNA3 (*P* = 0.0482) showed the opposite trend. The mRNA expression of the other EPHA/EFNA family members was not significantly associated with nodal status. ER- and PR-negative patients had higher levels of EPHA1 (*P* < 0.0001), EPHA2 (*P* < 0.0001), EPHA4 (*P* < 0.0001), EPHA7 (*P* < 0.0001 and =0.0046, respectively), EFNA3 (*P* < 0.0001), EFNA4 (*P* < 0.0001), and EFNA5 (*P* < 0.0001). On the other hand, EPHA3 (*P* < 0.0001), EPHA6 (*P* < 0.0015 and =0.0066, respectively), and EFNA1 (*P* < 0.0001) were higher in ER- and PR-positive patients. The EPHA10 mRNA level was higher in ER-positive patients (*P* < 0.0001) but not significantly associated with PR status (*P* = 0.5102). EPHA5 mRNA expression was not significantly associated with ER (*P* = 0.2271) and PR (*P* = 0.2851) status. EPHA1, EPHA2, EFNA3, and EFNA4 (*P* < 0.0001, all) mRNA levels were significantly higher in the HER2-positive group than in the HER2-negative group. Only EPHA6 (*P* = 0.0031) and EFNA1 (*P* < 0.0001) were significantly increased in the HER2-negative group. The mRNA expression of the other EPHA/EFNA family members was not associated with HER2 status. Triple-negative status was positively correlated with the mRNA expression of EPHA1 (*P* < 0.0001), EPHA2 (*P* < 0.0001), EPHA4 (*P* < 0.0001), EPHA7 (*P* = 0.0002), EFNA3 (*P* < 0.0001), EFNA4 (*P* < 0.0001), and EFNA5 (*P* < 0.0001) and negatively correlated with EPHA3 (*P* < 0.0001) and EPHA10 (*P* = 0.0333). The mRNA expression of the other EPHA/EFNA family members was not associated with triple-negative status. P53 mutant status (sequence) was positively correlated with EPHA1, EPHA2, EFNA3, EFNA4, and EFNA5 (*P* < 0.0001 for all) and P53 wild-type status was positively correlated with EPHA3 (*P* < 0.0001), EPHA6 (*P* = 0.0035), and EFNA1 (*P* = 0.0206) mRNA expression. The mRNA expression of the other EPHA/EFNA family members was not associated with P53 mutant status.

### 3.4. Genetic Alterations of EPHA/EFNA in BrCa

Different kinds of genetic alterations, such as missense mutations, amplification, and deep deletions, regulate cancer-related gene expression and participate in oncogenesis. We speculated that genetic alterations may regulate the transcriptional levels of EPHA/EFNA. To investigate mutations and CNAs of the EPHA/EFNA family in BrCa, the OncoPrint feature of cBioPortal (http://www.cbioportal.org) was used to investigate the proportion and percentage of specimens with genetic alterations in EPHA/EFNA. The frequency of alterations in these genes among BrCa samples varied from 1.1% to 10% for individual genes as shown in Figure 3.

### 3.5. The Prognostic Value of EPHA/EFNA mRNA Expression in BrCa Patients

The prognostic value of the mRNA expression of 12 EPHA/EFNA family members in BrCa patients was examined using the Kaplan–Meier plotter. High mRNA expression of EPHA7 (Figure 4(g), HR = 1.49, 95% CI: 1.09–2.05, *P* = 0.012) and EFNA4 (Figure 4(k), HR = 1.31, 95% CI: 1.04–1.64, *P* = 0.02) was associated with poor OS. EPHA6 mRNA expression (Figure 4(f), HR = 1.34, 95% CI: 0.98–1.84, *P* = 0.067) was moderately associated with poor OS. High mRNA expression of EPHA3 (Figure 4(c), HR = 0.71, 95% CI: 0.57–0.89, *P* = 0.0023) and EPHA4 (Figure 4(d), HR = 0.72, 95% CI: 0.52–0.99, *P* = 0.045) was significantly associated with better OS. The mRNA expression levels of the other EPHA/EFNA family members were not significantly correlated with OS.

Regarding RFS, high mRNA expression of EPHA7 (Figure 5(g), HR = 1.21, 95% CI: 1.04–1.42, *P* = 0.014), EFNA3 (Figure 5(j), HR = 1.17, 95% CI: 1.04–1.33, *P* = 0.01), and EFNA4 (Figure 5(k), HR = 1.28, 95% CI: 1.14–1.44, *P* < 0.0001) was associated with worse RFS. High mRNA expression of other EPHA/EFNA family members was significantly associated with better RFS except EFNA1. The RFS curves are shown in Figure 5 (EPHA1: HR = 0.68, 95% CI: 0.61–0.76, *P* < 0.0001; EPHA2: HR = 0.8, 95% CI: 0.72–0.89, *P* < 0.0001; EPHA3: HR = 0.78, 95% CI: 0.7–0.87, *P* < 0.0001; EPHA4: HR = 0.74, 95% CI: 0.62–0.87, *P* = 0.00036; EPHA5: HR = 0.72, 95% CI: 0.61–0.86, *P* = 0.00019; EPHA6: HR = 0.82, 95% CI: 0.69–0.97, *P* = 0.019; EPHA10: HR = 0.61, 95% CI: 0.52–0.71, *P* < 0.0001; and EFNA5: HR = 0.74, 95% CI: 0.66–0.82, *P* < 0.0001).

### 3.6. The Prognostic Value of EPHA/EFNA mRNA Expression in BrCa Patients with Different Subtypes

To further analyze the effect of EPHA/EFNA according to the BrCa subtype, the prognostic value of EPHA/EFNA family members was assessed in BrCa patients with different molecular subtypes, including basal-like, luminal A, luminal B, and HER2+ subtypes according to the 2011 St. Gallen criteria [30]. Because OS data were lacking for some patients, this analysis was limited to RFS. In the basal-like subtype, high mRNA expression of EFNA1 (HR = 1.36, 95% CI: 1.06–1.76, *P* = 0.016) and EFNA4 (HR = 1.53, 95% CI: 1.16–2.01, *P* = 0.022) predicted an unfavorable RFS, whereas high mRNA expression levels of EPHA1 (HR = 0.61, 95% CI: 0.48–0.79, *P* = 0.0001), EPHA4 (HR = 0.69, 95% CI: 0.49–0.96, *P* = 0.0029), EPHA5 (HR = 0.45, 95% CI: 0.29–0.68, *P* = 0.00015), EPHA7 (HR = 0.68, 95% CI: 0.49–0.95, *P* = 0.022), and EFNA5 (HR = 0.69, 95% CI: 0.54–0.89, *P* = 0.0037) were correlated with better RFS. The remaining EPHA/EFNA members were not associated with prognosis in basal-like BrCa. (Table 2).

In the luminal A subtype, high mRNA expression levels of EPHA1 (HR = 0.63, 95% CI: 0.53–0.75, *P* < 0.0001), EPHA2 (HR = 0.61, 95% CI:0.51–0.72, *P* < 0.0001), EPHA3 (HR = 0.73, 95% CI: 0.61–0.87, *P* = 0.00046), EPHA4 (HR = 0.69, 95% CI: 0.54–0.88, *P* = 0.0026), EPHA10 (HR = 0.54, 95% CI: 0.42–0.7, *P* < 0.0001), EFNA3 (HR = 0.81, 95% CI: 0.68–0.96, *P* = 0.017), EFNA4 (HR = 0.72, 95% CI: 0.6–0.86, *P* = 0.00036), and EFNA5 (HR = 0.61, 95% CI: 0.51–0.73, *P* < 0.0001) were associated with better RFS, whereas the high mRNA expression level of EPHA7 (HR = 1.49, 95% CI: 1.16–1.91, *P* = 0.0016) was associated with unfavorable RFS. The remaining EPHA/EFNA members were not associated with prognosis in luminal A BrCa.

In the luminal B subtype, high mRNA expression levels of EPHA1 (HR = 0.63, 95% CI: 0.52–0.76, *P* < 0.0001), EPHA2 (HR = 0.76, 95% CI: 0.63–0.93, *P* = 0.0067), EPHA4 (HR = 0.57, 95% CI: 0.42–0.79, *P* = 0.00047), EPHA5 (HR = 0.66, 95% CI: 0.48–0.89, *P* = 0.0068), EPHA6 (HR = 0.61, 95% CI: 0.45–0.85, *P* = 0.0026), EPHA10 (HR = 0.55, 95% CI: 0.4–0.75, *P* = 0.00012), and EFNA5 (HR = 0.67, 95% CI: 0.55–0.83, *P* = 0.00015) were associated with better RFS, whereas high mRNA expression levels of EFNA1 (HR = 1.38, 95% CI: 1.09–1.75, *P* = 0.0065), EFNA3 (HR = 1.39, 95% CI: 1.1–1.76, *P* = 0.0057), and EFNA4 (HR = 1.29, 95% CI: 1.05–1.6, *P* = 0.016) were associated with worse RFS. The remaining EPHA/EFNA members were not associated with prognosis in luminal B BrCa.

In HER2+ BrCa patients, high mRNA expression levels of EPHA1 (HR = 0.55, 95% CI: 0.37–0.8, *P* = 0.0019), EPHA6 (HR = 0.53, 95% CI: 0.29–0.94, *P* = 0.028), and EFNA5 (HR = 0.66, 95% CI: 0.45–0.97, *P* = 0.033) were correlated with better RFS. Only high mRNA expression of EPHA7 (HR = 2.32, 95% CI: 1.45–3.72, *P* = 0.00031) was associated with worse RFS. The remaining EPHA/EFNA members were not associated with prognosis in HER2-overexpressing BrCa. These results indicate that EPHA/EFNA may serve as potential prognostic predictors in BrCa patients with different subtype.

### 3.7. The Prognostic Value of EPHA/EFNA mRNA Expression in BrCa Patients Treated with Chemotherapy

The prognostic value of EPHA/EFNA expression was analyzed in BrCa patients receiving different chemotherapy regimens, including adjuvant chemotherapy, neoadjuvant chemotherapy, and no chemotherapy. As shown in Table 3, high expression of EPHA2 (HR = 1.49, 95% CI: 1.08–2.06, *P* = 0.016), EPHA3 (HR = 1.55, 95% CI: 1.12–2.15, *P* = 0.008), EPHA4 (HR = 1.95, 95% CI: 1.2–3.18, *P* = 0.0064), EFNA3 (HR = 1.96, 95% CI: 1.44–2.65, *P* < 0.001), and EFNA4 (HR = 1.4, 95% CI: 1.02–1.93, *P* = 0.037) and low expression of EPHA5 (HR = 0.43, 95% CI: 0.25–0.93, *P* = 0.002), EPHA6 (HR = 0.51, 95% CI: 0.27–0.95, *P* = 0.03), and EPHA10 (HR = 0.48, 95% CI: 0.29–0.8, *P* = 0.0043) were significantly correlated with poor RFS in BrCa patients treated with adjuvant chemotherapy. High expression levels of EPHA3 (HR = 1.95, 95% CI: 1–3.8, *P* = 0.048) and EPHA10 (HR = 2.43, 95% CI: 1.16–5.9, *P* = 0.016) and low expression of EPHA1 (HR = 0.39, 95% CI: 0.22–0.68, *P* < 0.001), EPHA2 (HR = 0.55, 95% CI: 0.31–0.97, *P* = 0.037), and EPHA5 (HR = 0.34, 95% CI: 0.16–0.77, *P* = 0.004) were significantly correlated with poor RFS in BrCa patients treated with neoadjuvant chemotherapy. These results indicate that EPHA/EFNA may serve as potential prognostic factors in BrCa patients treated with chemotherapy, suggesting that these genes are potential targets for the treatment of BrCa.

## 4. Discussion

The activities of the EPHA/EFNA family in BrCa are complex and paradoxical. The expression and prognostic value of EPHA/EFNA in BrCa have not been extensively investigated. In the present study, two cancer databases were used to analyze the transcriptional levels of EPHA/EFNA family members in BrCa and paracancerous tissues, as well as their association with the BrCa subtype and clinicopathological features. The genetic alterations of EPHA/EFNA family members, including mutations and putative CNAs, were analyzed using cBioPortal. The Kaplan–Meier plotter was used to analyze the association between the expression levels of EPHA/EFNA and OS or RFS in BrCa patients, as well as RFS in different BrCa subtypes, including patients undergoing chemotherapy. The results may be valuable in identifying new BrCa biomarkers for predicting prognosis or sensitivity to chemotherapy and suggest that EPHA and EFNA play both oncogenic and tumor suppressor roles in BrCa.

Expression analysis showed that the transcriptional levels of EPHA2, EPHA4, and EPHA5 were significantly lower in BrCa tissues than in nontumor tissues and EPHA1 and EPHA10 were significantly upregulated in BrCa tissues. Brantley et al. investigated EPHA/EFNA protein expression in BrCa and found that EPHA2, EPHA4, and EPHA7 were significantly upregulated in BrCa samples relative to normal controls. The discrepancy between the protein and mRNA levels of EPHA2 may be due to the fact that high levels of EPHA2 in tumor cells are the result of increased protein stability [31]. In certain malignant breast cell models, EPHA2 protein levels are 50- to 500-fold higher despite comparable levels of EphA2 mRNA [32, 33]. Discrepancies in EPHA2 expression may also result from the inclusion of both invasive and noninvasive breast tumors in the TCGA database. The mRNA level of EPHA2 is higher in invasive tumors than in normal breast cells; however, EPHA2 expression is lower in noninvasive breast tumors than in normal breast cells [34]. In this study, EFNA was upregulated in BrCa tissues except for EFNA5. EPHA2 is the dominant and the best characterized EPHA receptor in the BrCa. The role of EPHA2 in breast tumor progression is controversial, and conflicting data on the clinical significance of EPHA2 have been reported in different studies [35, 36]. For example, data show that EPHA2 is overexpressed in BrCa clinical samples; however, there is also evidence that EPHA2 acts as a tumor suppressor in breast carcinogenesis [17]. The malignant behavior of EPHA2 is mediated by ligand-independent signaling, and its antioncogenic properties are attributed to ligand-dependent signaling [37]. The crosstalk between EphA2 and BrCa oncogenic pathways promotes tumor cell malignancy in ligand-independent signaling [38, 39]. We found an inverse correlation between EPHA2 and the mRNA expression of A-type ligands in the database, as shown by the downregulation of EPHA2 and EFNA overexpression in BrCa cells. Ligand upregulation in the tumor indicates that the ligand-dependent pathway is dominant in the database. Downregulation of the EPHA2 receptor by the ephrin ligand may involve ligand-mediated receptor internalization. In general, EPHA2 negatively regulates tumor growth and migration after canonical ligand-induced EPHA2 signaling, which inhibits the AKT-mTORC1 and MAPK pathways [17]. The interaction between EPHA2 and its ligand activates a negative feedback pathway mediated by growth factor-activated RAS signaling [40]. EFNA1 is upregulated in noninvasive breast cells, thereby inhibiting invasiveness, whereas EFNA1 is downregulated in invasive tumors, allowing EPHA2 to participate in invasion [34].

We also compared the differential transcriptional levels of EPHA/EFNA family members according to the different intrinsic subtypes of BrCa. The results showed differences in the expression patterns between the BrCa subtypes. EPHA3, EPHA5, EPHA6, and EPHA10 were expressed at the highest levels in luminal tissues, whereas HER2-positive and triple-negative tissues tended to express lower levels of EPHA3, EPHA5, EPHA6, and EPHA10. The highest mRNA expression levels of EFNA were found in triple-negative tissues except EFNA3, whereas the lowest mRNA expression levels of EFNA were found in the luminal subtype except EFNA1. Analysis of the bc-GenExMiner database showed that EPHA1, EPHA2, EPHA4, EPHA7, EFNA3, EFNA4, and EFNA5 were upregulated in ER- and PR-negative patients and positively correlated with triple-negative status. Consistent with this, some studies have shown that EPHA2 overexpression in BrCa is negatively correlated with ER and PR status [32, 41, 42]. EPHA2 overexpression decreases estrogen dependence and tamoxifen sensitivity [43], and EPHA2 is preferentially expressed in the basal-like phenotype [44]. In contrast, EPHA2 expression is also negatively regulated by ER*α* [41] and wild-type p53 [45]. The correlation of EPHA2 with HER2-positive status in the present study is consistent with the results of previous studies [39, 46], and EPHA2 is associated with resistance to trastuzumab therapy [47].

Analysis of the other EPHA/EFNA family members showed that EPHA1 was significantly upregulated in BrCa tissues compared to paracancerous tissues. A previous report showed that EPHA1 downregulation is associated with the invasiveness of breast carcinoma cells [34]. Consistent with the present profiling analyses, EPHA4 expression is associated with basal-like BrCa [48] and EPHA5 has been reported to act as a tumor suppressor, which may be related to abrrant promoter methylation [49]. Liu et al. [50] showed that EPHA7 mRNA was downregulated in BrCa specimens and loss of EPHA7 expression is more common in high-grade, early TNM-stage patients, without lymph node metastasis and correlation with negative HER2 status. Correspondingly, the present data also found downregulation of EPHA7 expression in BrCa specimens. EPHA10 is the only kinase-deficient Eph receptor [51]. The present data indicate that EPHA10 is upregulated in BrCa tissues, which is similar with a previous study showing that EPHA10 expression is significantly lower in invasive than in noninvasive breast tumors, and is absent in normal cells [34]. Similar with the previous study, the present data showed EFNA4 was upregulated in TNBC [52]. EFNA4 is required for proper differentiation and polarization of mammary epithelial cells, signifying a biologic basis for the overexpression of EFNA4 in BrCa [53].

The most common cancer-related genetic alteration is the DNA CNAs. The OncoPrint feature of cBioPortal was used to determine the frequency of genetic alterations in the EPHA/EFNA family. The results showed that EPHA/EFNA was not frequently amplified. This finding suggests that the EPHA/EFNA family does not affect BrCa survival through DNA alterations, whereas it may affect BrCa through alterations of the interaction network. The copy-gain frequency of EFNA1, EFNA3, and EFNA4 accounts for a large proportion of BrCa samples, which may explain the significant upregulation of EFNA1, EFNA3, and EFNA4 in BrCa tissues from UALCAN.

The Kaplan–Meier plotter is a survey of public microarray data repositories of survival from 3955 patients with BrCa. Besides, in general patients, we analyzed the prognostic value of EPHA/EFNA mRNA in different BrCa subtypes and in BrCa patients treated with chemotherapy. Large-scale expression profiling studies revealed a negative association between the overexpression of EPHA2, EPHA4, and EPHA7 and overall and disease-free survival in BrCa [54]. Consistent with this report and its positive correlation with the triple-negative (TNBC) status in the bc-GenExMiner, the Kaplan–Meier plotter indicated that high EPHA7 mRNA expression predicted a poor OS and RFS in BrCa, especially in the HER2+ and luminal A subtypes. EFNA4 was associated with poor OS and RFS in BrCa, which is consistent with its positive correlation with the TNBC status. In particular, EFNA4 was associated with poor RFS in luminal B and basal-like subtypes and in BrCa patients treated with adjuvant chemotherapy. High mRNA expression of EPHA3 was significantly associated with better OS and RFS, especially in the luminal A subtype, which is consistent with its negative correlation with the TNBC status. However, in patients receiving adjuvant chemotherapy and neoadjuvant chemotherapy, EPHA3 is a risk factor. These results suggest that EPHA3, EPHA7 and EFNA4 are involved in BrCa development and could predict the prognosis of patients with BrCa in various subtypes and in those receiving different chemotherapy regimens. BrCa is a heterogeneous disease with subtype-dependent histopathological and clinical significance. In the subgroup analysis, the triple-negative (basal-like) subtype is a unique subtype of BrCa with a poor prognosis and more likely to develop chemoresistance [55]. In this study, we showed that low expression of EPHA1, EPHA4, EPHA5, and EPHA7 and high expression of EFNA1, EFNA4, and EFNA5 predicted an unfavorable prognosis in basal-like patients. Although we found that high mRNA expression of EPHA2 was associated with a longer RFS in patients with BrCa, it was a risk factor in the cohort receiving adjuvant chemotherapy. In fact, the RSK1/2-EphA2-GPRC5A oncogenic signaling association with platinum chemotherapy resistance has been reported in recent study [19] . Furthermore, in clinical practice, these biomarkers coupled with the specific role of EPHA/EFNA signaling in cancer could promote targeted therapeutics, as reported before [52, 56].

The present study has several limitations that should be addressed in future studies. First, mRNA levels are not always indicative of a functional protein and thus may not fully represent the protein expression of EPHA/EFNA [25]. Future studies should include protein detection techniques to accurately assess the protein levels. Second, the function of EPHA3 and EFNA7 in BrCa has not been studied in BrCa and needs to be investigated in the future. Third, multivariate analysis could not be used in the database to correct the associations between different clinicopathological features.

In conclusion, we showed that the EPHA/EFNA family is widely expressed in BrCa tumor cells. EPHA/EFNA were identified as prognostic factors and potential targets for BrCa, which may improve our understanding of the complexity and heterogeneity of BrCa at the molecular level. The present results may help develop tools to accurately predict prognosis and design customized therapies.

## Figures and Tables

**Figure 1:** Transcriptional levels of EPHA/EFNA in breast cancer and paracancerous tissues from the TCGA dataset based on data mining via UALCAN. The transcriptional levels of EPHA1, EPHA10, EFNA1, EFNA3, and EFNA4 (a, h, i, j, and k) were upregulated, whereas the transcriptional levels of EPHA2, EPHA4, EPHA5, and EFNA5 (b, d, e, and l) were downregulated in breast cancer tissues compared with paracancerous tissues. The transcriptional levels of EPHA3, EPHA6, and EPHA7 (c, f, and g) did not differ significantly between breast cancer and paracancerous tissues.

**Figure 2:** The transcriptional level of EPHA/EFNA in breast cancer patients with different subtypes. HER2-positive and triple-negative breast cancer patients tended to express lower levels of EPHA3, EPHA5, EPHA6, and EPHA10 mRNA. The highest mRNA expression of EPHA3, EPHA5, EPHA6, and EPHA10 was found in the luminal subtype. The highest mRNA expression of EFNA was detected in triple-negative tissues except EFNA3, and the lowest mRNA expression of EFNA was detected in the luminal subtype, except for EFNA1.

**Figure 3:** EPHA/EFNA family gene alteration analysis in invasive breast carcinoma. OncoPrint represents the distribution and percentages of samples with different types of alterations in the EPHA/EFNA family. The right part of the figure without alterations was not included.

**Figure 4:** Survival analyses of EPHA/EFNA in breast cancer (overall survival (OS) in the Kaplan–Meier plotter). High mRNA expression of EPHA7 (g) and EFNA4 (k) was associated with poor OS. EPHA6 (f) expression was moderately associated with poor OS. High mRNA expression of EPHA3 (c) and EPHA4 (d) was significantly associated with better OS. The mRNA expression levels of the other EPHA/EFNA family members were not significantly correlated with OS.

**Figure 5:** Survival analyses of the EPHA/EFNA in breast cancer (recurrence-free survival (RFS) in the Kaplan–Meier plotter). High mRNA expression of EPHA7 (g), EFNA3 (j) and EFNA4 (k) was associated with worse RFS. High mRNA expression of other EPHA/EFNA family members was significantly associated with better RFS except EFNA1.

**(a):** 

Parameters	EPHA1	EPHA2	EPHA3	EPHA4	EPHA5	EPHA6
Age (years)	0.2250			0.3583	0.8373	0.1242
>51						
≤51		0.0002	<0.0001			
Nodal status	0.9075		0.6126	0.5222	0.9379	0.2129
Negative		0.0142				
Positive						
ER (IHC)					0.2271	
Negative	<0.0001	<0.0001		<0.0001		
Positive			<0.0001			0.0015
PR (IHC)					0.2851	
Negative	<0.0001	<0.0001		<0.0001		
Positive			<0.0001			0.0066
HER2 (IHC)			0.1385	0.7082	0.4015	
Negative						0.0031
Positive	<0.0001	<0.0001				
Triple-negative status					0.0924	0.4042
Not			<0.0001			
TNBC	<0.0001	<0.0001		<0.0001		
P53 sequence				0.2714	0.5513	
Wild type			<0.0001			0.0035
Mutated	<0.0001	<0.0001				

**(b):** 

Parameters	EPHA7	EPHA10	EFNA1	EFNA3	EFNA4	EFNA5
Age (years)	0.0577	0.0878				
>51			<0.0001	0.0092		
≤51					0.0003	<0.0001
Nodal status	0.9157	0.7342	0.4045		0.6819	0.7867
Negative						
Positive				0.0482		
ER (IHC)						
Negative	<0.0001			<0.0001	<0.0001	<0.0001
Positive		<0.0001	<0.0001			
PR (IHC)		0.5102				
Negative	0.0046			<0.0001	<0.0001	<0.0001
Positive			<0.0001			
HER2 (IHC)	0.9010	0.9299				0.5285
Negative			<0.0001			
Positive				<0.0001	<0.0001	
Triple-negative status			0.3715			
Not		0.0333				
TNBC	0.0002			<0.0001	<0.0001	<0.0001
P53 sequence	0.4840	0.1113				
Wild type			0.0206			
Mutated				<0.0001	<0.0001	<0.0001

**Table 2:** Prognostic values of EPHA/EFNA mRNA expression for RFS in different BrCa intrinsic subtypes.

Subclasses	*N*	HR (95% CI)	*P*
EPHA1			
Basal like	618	0.61 (0.48–0.79)	0.0001
Luminal A	1,933	0.63 (0.53–0.75)	<0.0001
Luminal B	1,149	0.63 (0.52–0.76)	<0.0001
HER2 positive	251	0.55 (0.37–0.8)	0.0019
EPHA2			
Basal like	618	0.84 (0.65–1.09)	0.19
Luminal A	1,933	0.61 (0.51–0.72)	<0.0001
Luminal B	1,149	0.76 (0.63–0.93)	0.0067
HER2 positive	251	0.669 (0.42-1.03)	0.068
EPHA3			
Basal like	618	0.85 (0.65–1.11)	0.23
Luminal A	1,933	0.73 (0.61–0.87)	0.00046
Luminal B	1,149	1.21 (0.96–1.52)	0.1
HER2 positive	251	0.74 (0.5–1.08)	0.11
EPHA4			
Basal like	360	0.69 (0.49–0.96)	0.029
Luminal A	841	0.69 (0.54–0.88)	0.0026
Luminal B	407	0.57 (0.42–0.79)	0.00047
HER2 positive	156	0.74 (0.46–1.18)	0.21
EPHA5			
Basal like	360	0.45 (0.29–0.68)	0.00015
Luminal A	841	0.77 (0.59–1.01)	0.059
Luminal B	407	0.66 (0.48–0.89)	0.0068
HER2 positive	156	0.74 (0.46–1.19)	0.21
EPHA6			
Basal like	360	0.78 (0.53–1.15)	0.21
Luminal A	841	1.18 (0.91–1.52)	0.21
Luminal B	407	0.61 (0.45–0.85)	0.0026
HER2 positive	156	0.53 (0.29–0.94)	0.028
EPHA7			
Basal like	360	0.68 (0.49–0.95)	0.022
Luminal A	841	1.49 (1.16–1.91)	0.0016
Luminal B	407	0.84 (0.61–1.15)	0.27
HER2 positive	156	2.32 (1.45–3.72)	0.00031
EPHA10			
Basal like	360	0.71 (0.49–1.02)	0.064
Luminal A	841	0.54 (0.42–0.7)	<0.0001
Luminal B	407	0.55 (0.4–0.75)	0.00012
HER2 positive	156	1.28 (0.75–2.2)	0.37
EFNA1			
Basal like	618	1.36 (1.06–1.76)	0.016
Luminal A	1,933	0.89 (0.73–1.07)	0.21
Luminal B	1,149	1.38 (1.09–1.75)	0.0065
HER2 positive	251	1.45 (0.91–2.33)	0.12
EFNA3			
Basal like	618	1.29 (0.97–1.73)	0.082
Luminal A	1,933	0.81 (0.68–0.96)	0.017
Luminal B	1,149	1.39 (1.1–1.76)	0.0057
HER2 positive	251	1.43 (0.96–2.14)	0.081
EFNA4			
Basal like	618	1.53 (1.16–2.01)	0.0022
Luminal A	1,933	0.72 (0.6–0.86)	0.00036
Luminal B	1,149	1.29 (1.05–1.6)	0.016
HER2 positive	251	0.82 (0.51–1.3)	0.39
EFNA5			
Basal like	618	0.69 (0.54–0.89)	0.0037
Luminal A	1,933	0.61 (0.51–0.73)	<0.0001
Luminal B	1,149	0.67 (0.55–0.83)	0.00015
HER2 positive	251	0.66 (0.45–0.97)	0.033

**Table 3:** Prognostic value of EPHA/EFNA mRNA expression for RFS in BrCa patients undergoing chemotherapy.

Chemotherapies	Cases of RFS	HR	95% CI	*P* value
EPHA1				
Adjuvant chemotherapy	594	1.28	0.94–1.73	0.11
Neoadjuvant chemotherapy	223	0.39	0.22–0.68	<0.001
Nonchemotherapy	1,873	0.82	0.69–0.97	0.023
EPHA2				
Adjuvant chemotherapy	594	1.49	1.08–2.06	0.016
Neoadjuvant chemotherapy	223	0.55	0.31–0.97	0.037
Nonchemotherapy	1,873	0.8	0.66–0.98	0.029
EPHA3				
Adjuvant chemotherapy	594	1.55	1.12–2.15	0.008
Neoadjuvant chemotherapy	223	1.95	1–3.8	0.048
Nonchemotherapy	1,873	0.71	0.58–0.87	0.001
EPHA4				
Adjuvant chemotherapy	255	1.95	1.2–3.18	0.0064
Neoadjuvant chemotherapy	111	0.76	0.35–1.65	0.48
Nonchemotherapy	243	1.57	0.91–2.71	0.1
EPHA5				
Adjuvant chemotherapy	255	0.43	0.25–0.93	0.002
Neoadjuvant chemotherapy	111	0.34	0.16–0.77	0.004
Nonchemotherapy	243	0.69	0.39–1.22	0.2
EPHA6				
Adjuvant chemotherapy	255	0.51	0.27–0.95	0.03
Neoadjuvant chemotherapy	111	1.9	0.9–3.99	0.086
Nonchemotherapy	243	0.7	0.39–1.24	0.22
EPHA7				
Adjuvant chemotherapy	255	0.64	0.4–1.03	0.065
Neoadjuvant chemotherapy	111	1.86	0.82–4.23	0.13
Nonchemotherapy	243	1.42	0.82–2.46	0.21
EPHA10				
Adjuvant chemotherapy	255	0.48	0.29–0.8	0.0043
Neoadjuvant chemotherapy	111	2.43	1.16–5.9	0.016
Nonchemotherapy	243	0.62	0.35–1.11	0.1
EFNA1				
Adjuvant chemotherapy	594	0.82	0.6–1.11	0.2
Neoadjuvant chemotherapy	223	0.73	0.42–1.26	0.25
Nonchemotherapy	1,873	0.82	0.69–0.97	0.02
EFNA3				
Adjuvant chemotherapy	594	1.96	1.44–2.65	<0.001
Neoadjuvant chemotherapy	223	1.34	0.77–2.32	0.3
Nonchemotherapy	1,873	1.2	1–1.44	0.05
EFNA4				
Adjuvant chemotherapy	594	1.4	1.02–1.93	0.037
Neoadjuvant chemotherapy	223	0.71	0.41–1.23	0.22
Nonchemotherapy	1,873	0.86	0.73–1.02	0.077
EFNA5				
Adjuvant chemotherapy	594	0.85	0.6–1.19	0.34
Neoadjuvant chemotherapy	223	0.63	0.35–1.14	0.12
Nonchemotherapy	1,873	0.78	0.64–0.95	0.012

## Data Availability

The data used to support the findings of this study are included within the article.

## Abbreviations

EPHA: Ephrin A
HR: Hazard ratio
BrCa: Breast cancer
KM plotter: Kaplan–Meier plotter
RFS: Relapse-free survival
RTK: Tyrosine kinase receptor
CI: Confidence interval
ER: Estrogen receptor
PR: Progesterone receptor
HER2: Human epidermal growth factor receptor 2
SPSS: Statistical product and service solutions
OS: Overall survival.

## References

[1] Sung H., Ferlay J., Siegel R., Soerjomataram I., Jemal A., Bray F. (2021). Global cancer statistics 2020: GLOBOCAN estimates of incidence and mortality worldwide for 36 cancers in 185 countries. *CA: a Cancer Journal for Clinicians*.

[2] Berry D. A., Cronin K. A., Plevritis S. K. (2005). Effect of screening and adjuvant therapy on mortality from breast cancer. *The New England Journal of Medicine*.

[3] Du Z., Lovly C. M. (2018). Mechanisms of receptor tyrosine kinase activation in cancer. *Molecular Cancer*.

[4] Lisabeth E. M., Falivelli G., Pasquale E. B. (2013). Eph receptor signaling and ephrins. *Cold Spring Harbor Perspectives in Biology*.

[5] Pasquale E. B. (2008). Eph-ephrin bidirectional signaling in physiology and disease. *Cell*.

[6] Eph Nomenclature Committee (1997). Unified nomenclature for Eph family receptors and their ligands, the ephrins. *Cell*.

[7] Pasquale E. B. (2010). Eph receptors and ephrins in cancer: bidirectional signalling and beyond. *Nature Reviews. Cancer*.

[8] Kou C.-T. J., Kandpal R. P. (2018). Differential expression patterns of Eph receptors and Ephrin ligands in human cancers. *BioMed Research International*.

[9] Mosch B., Reissenweber B., Neuber C., Pietzsch J. (2010). Eph receptors and ephrin ligands: important players in angiogenesis and tumor angiogenesis. *Journal of Oncology*.

[10] Easty D. J., Hill S. P., Hsu M. Y. (1999). Up-regulation of ephrin-A1 during melanoma progression. *International Journal of Cancer*.

[11] Walker-Daniels J., Coffman K., Azimi M. (1999). Overexpression of the EphA2 tyrosine kinase in prostate cancer. *Prostate*.

[12] Xiang Y.-P., Xiao T., Li Q. G. (2020). Y772 phosphorylation of EphA2 is responsible for EphA2-dependent NPC nasopharyngeal carcinoma growth by Shp2/Erk-1/2 signaling pathway. *Cell Death & Disease*.

[13] Liu Y., Zhang X., Qiu Y. (2011). Clinical significance of EphA2 expression in squamous-cell carcinoma of the head and neck. *Journal of Cancer Research and Clinical Oncology*.

[14] Govindan R., Ding L., Griffith M. (2012). Genomic landscape of non-small cell lung cancer in smokers and never-smokers. *Cell*.

[15] Oricchio E., Nanjangud G., Wolfe A. L. (2011). The Eph-receptor A7 is a soluble tumor suppressor for follicular lymphoma. *Cell*.

[16] Walker-Daniels J., Hess A. R., Hendrix M. J. C., Kinch M. S. (2003). Differential regulation of EphA2 in normal and malignant cells. *The American Journal of Pathology*.

[17] Noblitt L. W., Bangari D. S., Shukla S. (2004). Decreased tumorigenic potential of EphA2-overexpressing breast cancer cells following treatment with adenoviral vectors that express EphrinA1. *Cancer Gene Therapy*.

[18] Wang Y., Liu Y., Li G. (2015). Ephrin type-A receptor 2 regulates sensitivity to paclitaxel in nasopharyngeal carcinoma via the phosphoinositide 3-kinase/Akt signalling pathway. *Molecular Medicine Reports*.

[19] Moyano-Galceran L., Pietilä E. A., Turunen S. P. (2020). Adaptive RSK-EphA2-GPRC5A signaling switch triggers chemotherapy resistance in ovarian cancer. *EMBO Molecular Medicine*.

[20] Barrett T., Wilhite S. E., Ledoux P. (2012). NCBI GEO: archive for functional genomics data sets—update. *Nucleic Acids Research*.

[21] The Cancer Genome Atlas Research Network, Weinstein J. N., Collisson E. A. (2013). The Cancer Genome Atlas Pan-Cancer analysis project. *Nature Genetics*.

[22] Chandrashekar D. S., Bashel B., Balasubramanya S. A. H. (2017). UALCAN: a portal for facilitating tumor subgroup gene expression and survival analyses. *Neoplasia*.

[23] Jézéquel P., Campone M., Gouraud W. (2012). bc-GenExMiner: an easy-to-use online platform for gene prognostic analyses in breast cancer. *Breast Cancer Research and Treatment*.

[24] Jezequel P., Frenel J. S., Campion L. (2013). bc-GenExMiner 3.0: new mining module computes breast cancer gene expression correlation analyses. *Database*.

[25] Mei J., Hao L., Liu X. (2019). Comprehensive analysis of peroxiredoxins expression profiles and prognostic values in breast cancer. *Biomarker Research*.

[26] Györffy B., Lanczky A., Eklund A. C. (2010). An online survival analysis tool to rapidly assess the effect of 22,277 genes on breast cancer prognosis using microarray data of 1,809 patients. *Breast Cancer Research and Treatment*.

[27] Cerami E., Gao J., Dogrusoz U. (2012). The cBio cancer genomics portal: an open platform for exploring multidimensional cancer genomics data. *AACR.*.

[28] Gao J., Aksoy B. A., Dogrusoz U. (2013). Integrative analysis of complex cancer genomics and clinical profiles using the cBioPortal. *Science Signaling*.

[29] Goto W., Kashiwagi S., Takada K. (2018). Significance of intrinsic breast cancer subtypes on the long-term prognosis after neoadjuvant chemotherapy. *Journal of Translational Medicine*.

[30] Goldhirsch A., Wood W. C., Coates A. S. (2011). Strategies for subtypes--dealing with the diversity of breast cancer: highlights of the St Gallen International Expert Consensus on the Primary Therapy of Early Breast Cancer 2011. *Annals of Oncology*.

[31] Walker-Daniels J., Riese D. J., Kinch M. S. (2002). c-Cbl-dependent EphA2 protein degradation is induced by ligand binding. *Molecular Cancer Research*.

[32] Zelinski D. P., Zantek N. D., Stewart J. C., Irizarry A. R., Kinch M. S. (2001). EphA2 overexpression causes tumorigenesis of mammary epithelial cells. *Cancer Research*.

[33] Zantek N. D., Walker-Daniels J., Stewart J. (2001). MCF-10A-NeoST: a new cell system for studying cell-ECM and cell-cell interactions in breast cancer. *Clinical Cancer Research*.

[34] Fox B. P., Kandpal R. P. (2004). Invasiveness of breast carcinoma cells and transcript profile: Eph receptors and ephrin ligands as molecular markers of potential diagnostic and prognostic application. *Biochemical and Biophysical Research Communications*.

[35] Pan M. (2005). Overexpression ofEphA2gene in invasive human breast cancer and its association with hormone receptor status. *Journal of Clinical Oncology*.

[36] Ogawa K., Pasqualini R., Lindberg R. A., Kain R., Freeman A. L., Pasquale E. B. (2000). The ephrin-A1 ligand and its receptor, EphA2, are expressed during tumor neovascularization. *Oncogene*.

[37] Miao H., Li D. Q., Mukherjee A. (2009). EphA2 mediates ligand-dependent inhibition and ligand-independent promotion of cell migration and invasion via a reciprocal regulatory loop with Akt. *Cancer Cell*.

[38] Brantley-Sieders D. M., Zhuang G., Hicks D. (2008). The receptor tyrosine kinase EphA2 promotes mammary adenocarcinoma tumorigenesis and metastatic progression in mice by amplifying ErbB2 signaling. *The Journal of Clinical Investigation*.

[39] Zhuang G., Brantley-Sieders D., Hicks D., Fang W., Hwang Y., Chen J. (2008). Interactions of EphA2 and HER2 promote tumor progression and anti-HER2 resistance. *AACR.*.

[40] Macrae M., Neve R. M., Rodriguez-Viciana P. (2005). A conditional feedback loop regulates Ras activity through EphA2. *Cancer Cell*.

[41] Zelinski D. P., Zantek N. D., Walker-Daniels J., Peters M. A., Taparowsky E. J., Kinch M. S. (2002). Estrogen and Myc negatively regulate expression of the EphA2 tyrosine kinase. *Journal of Cellular Biochemistry*.

[42] Kamat A. A., Coffey D., Merritt W. M. (2009). EphA2 overexpression is associated with lack of hormone receptor expression and poor outcome in endometrial cancer. *Cancer*.

[43] Lu M., Miller K. D., Gokmen-Polar Y., Jeng M. H., Kinch M. S. (2003). EphA2 overexpression decreases estrogen dependence and tamoxifen sensitivity. *Cancer Research*.

[44] Huang F., Reeves K., Han X. (2007). Identification of candidate molecular markers predicting sensitivity in solid tumors to dasatinib: rationale for patient selection. *Cancer Research*.

[45] Dohn M., Jiang J., Chen X. (2001). Receptor tyrosine kinase EphA2 is regulated by p53-family proteins and induces apoptosis. *Oncogene*.

[46] Youngblood V. M., Kim L. C., Edwards D. N. (2016). The Ephrin-A1/EPHA2 signaling axis regulates glutamine metabolism in HER2-positive breast cancer. *Cancer Research*.

[47] Zhuang G., Brantley-Sieders D. M., Vaught D. (2010). Elevation of receptor tyrosine kinase EphA2 mediates resistance to trastuzumab therapy. *Cancer Research*.

[48] Hachim I. Y., Villatoro M., Canaff L. (2017). Transforming growth factor-beta regulation of ephrin type-A receptor 4 signaling in breast cancer cellular migration. *Scientific Reports*.

[49] Fu D. Y., Wang Z. M., Wang B. L. (2010). Frequent epigenetic inactivation of the receptor tyrosine kinase EphA5 by promoter methylation in human breast cancer. *Human Pathology*.

[50] Liu Z., Zhang Q., Li X., Tao Z. (2016). Aberrant expression of receptor tyrosine kinase EphA7 in breast cancers. *International Journal of Clinical and Experimental Pathology*.

[51] Murai K. K., Pasquale E. B. (2003). ‘Eph’ective signaling: forward, reverse and crosstalk. *Journal of Cell Science*.

[52] Damelin M., Bankovich A., Park A. (2015). Anti-EFNA4 calicheamicin conjugates effectively target triple-negative breast and ovarian tumor-initiating cells to result in sustained tumor regressions. *Clinical Cancer Research*.

[53] Burleigh A., McKinney S., Brimhall J. (2015). A co-culture genome-wide RNAi screen with mammary epithelial cells reveals transmembrane signals required for growth and differentiation. *Breast Cancer Research*.

[54] Brantley-Sieders D. M., Jiang A., Sarma K. (2011). Eph/ephrin profiling in human breast cancer reveals significant associations between expression level and clinical outcome. *PLoS One*.

[55] Boichuk S., Galembikova A., Sitenkov A. (2017). Establishment and characterization of a triple negative basal-like breast cancer cell line with multi-drug resistance. *Oncology Letters*.

[56] Lee J. W., Han H. D., Shahzad M. M. K. (2009). EphA2 immunoconjugate as molecularly targeted chemotherapy for ovarian carcinoma. *Journal of the National Cancer Institute*.

